The article "Statins dose-dependently exert a chemopreventive effect against lung cancer in COPD patients: a population-based cohort study" was published in 2016. Journal: Oncotarget.

# Statins dose-dependently exert a chemopreventive effect against lung cancer in COPD patients: a population-based cohort study

**DOI:** 10.18632/oncotarget.11162

**Published:** 2016-08-09

**Authors:** Ju-Chi Liu, Tsung-Yeh Yang, Yi-Ping Hsu, Wen-Rui Hao, Pai-Feng Kao, Li-Chin Sung, Chun-Chao Chen, Szu-Yuan Wu

**Affiliations:** ^1^ Division of Cardiovascular Medicine, Department of Internal Medicine, Shuang Ho Hospital, Taipei Medical University, New Taipei City, Taiwan; ^2^ Institute of Toxicology, College of Medicine, National Taiwan University, Taipei, Taiwan; ^3^ Department of Radiation Oncology, Wan Fang Hospital, Taipei Medical University, Taipei, Taiwan; ^4^ Department of Internal Medicine, School of Medicine, College of Medicine, Taipei Medical University, Taipei, Taiwan; ^5^ Department of Biotechnology, Hungkuang University, Taichung, Taiwan

**Keywords:** statins, COPD, lung cancer

## Abstract

**Purpose:**

Chronic obstructive pulmonary disease (COPD) is associated with increased lung cancer risk. We evaluated the association of statin use with lung cancer risk in COPD patients and identified which statins possess the highest chemopreventive potential.

**Results:**

After adjustment for age, sex, CCI, diabetes, hypertension, dyslipidemia, urbanization level, and monthly income according to propensity scores, lung cancer risk in the statin users was lower than that in the statin nonusers (adjusted hazard ratio [aHR] = 0.37). Of the individual statins, lovastatin and fluvastatin did not reduce lung cancer risk significantly. By contrast, lung cancer risk in patients using rosuvastatin, simvastatin, atorvastatin, and pravastatin was significantly lower than that in statin nonusers (aHRs = 0.41, 0.44, 0.52, and 0.58, respectively). Statins dose-dependently reduced lung cancer risk in all subgroups and the main model with additional covariates (nonstatin drug use).

**MATERIALS AND METHODS:**

The study cohort comprised all patients diagnosed with COPD at health care facilities in Taiwan (*n* = 116,017) between January 1, 2001 and December 31, 2012. Our final study cohort comprised 43,802 COPD patients: 10,086 used statins, whereas 33,716 did not. Patients were followed up to assess lung cancer risk or protective factors. In addition, we also considered demographic characteristics, namely age, sex, comorbidities (diabetes, hypertension, dyslipidemia, and Charlson comorbidity index [CCI]), urbanization level, monthly income, and nonstatin drug use. The index date of statin use was the COPD confirmation date. To examine the dose–response relationship, we categorized statin use into four groups in each cohort: < 28, 28–90, 91–365, and > 365 cumulative defined daily doses (cDDDs). Patients receiving < 28 cDDDs were defined as nonstatin users.

**Conclusions:**

Statins dose-dependently exert a significant chemopreventive effect against lung cancer in COPD patients. Rosuvastatin, simvastatin, and atorvastatin exhibited the highest chemopreventive potential.

## INTRODUCTION

Chronic obstructive pulmonary disease (COPD) is the seventh leading cause of death in Taiwan [1]. COPD is increasingly considered a multisystem disease characterized by both pulmonary and systemic inflammation. Comorbidities of COPD generally include diseases involving the pulmonary system (infective exacerbations, pneumonia, influenza, and lung cancer) and cardiovascular system (acute coronary syndrome, endothelial dysfunction, and pulmonary hypertension). COPD is independently associated with increased lung cancer risk, which is probably associated with the inflammation and scarring that occurs during COPD development [2–4]. Moreover, lung cancer is the leading cause of cancer death in Taiwan [1].

Our previous observational studies have suggested that statin use may reduce the overall risk of cancers and of specific cancers [5], possibly by inhibiting downstream products of the mevalonate pathway [6–9], triggering tumor-specific apoptosis [10], and inhibiting the proteasome pathway [11]. In theory, statins can reduce COPD-induced inflammation and scarring and further decrease lung cancer risk in patients with COPD. In addition, statins can reduce the risk of esophageal cancer [12], colorectal cancer [13], gastric cancer [14], hepatocellular carcinoma [15], and prostate cancer [16]. However, a meta-analysis indicated that statin use has no effect on lung cancer risk [17]. COPD and lung cancer are associated through several factors in addition to smoking or aeropollutant exposure [18–21]. Because patients with COPD have a high lung cancer risk, the effect of statins may differ from that observed previously [17].

Statins are the most powerful drugs available for reducing low-density lipoprotein cholesterol (LDL-C) levels; they are the most effective lipid-lowering drugs for improving clinical outcomes when used for the primary and secondary prevention of cardiovascular diseases. Statin selection depends upon several factors, including the degree of hyperlipidemia, pharmacokinetic properties of the drug, drug interactions, presence of renal impairment, and cost. Currently available statins include lovastatin, pravastatin, simvastatin, fluvastatin, atorvastatin, and rosuvastatin. These agents are competitive inhibitors of hydroxymethylglutaryl-coenzyme A (HMG-CoA) reductase, which is involved in the rate-limiting step of cholesterol biosynthesis. Statins occupy a portion of the HMG-CoA active site, blocking the binding of the substrate to the enzyme [22]. Most statins reduce LDL-C and triglycerides levels and moderately increase high-density lipoprotein cholesterol (HDL-C) levels; nevertheless, different statins have different efficacies. Whether these differences may be associated with a decrease in lung cancer risk remains unclear.

Thus, considering that systemic inflammation is implicated in lung cancer and that smoking- and obesity-related cancers may remain prevalent in the coming decades, we initiated this study targeting statin-based chemoprevention. Thus far, studies supporting the chemopreventive mechanism of statins against lung cancer in patients with COPD have been scant; in addition, variation in the chemoprevention profiles of individual statins is unclear. This is the first study to establish an association between statin use and the chemoprevention of lung cancer in patients with COPD, and is also the first study to investigate which statins exert the highest chemopreventive effects.

## RESULTS

Our COPD cohort comprised 43,802 patients, 10,086 (30%) of whom used statins and the remaining 33,716 (70%) of whom did not (Table 1). The total follow-up duration was 194,933.6 and 80,239.4 person-years for the statin nonusers and users, respectively. Compared with the statin nonusers, the statin users exhibited a higher prevalence of pre-existing medical comorbidities including diabetes, hypertension, and dyslipidemia, along with a higher CCI (all *P* < 0.001). In addition, significant differences were observed between the two groups in the distributions of age, monthly income, and urbanization level as well as use of nonstatin lipid-lowering drug, aspirin, ACEI, and metformin (Table 1). A higher proportion of statin nonusers used nonstatin lipid-lowering drugs, metformin, ACEI, and aspirin for < 28 days; however, most of the statin users used these drugs for > 365 days. A lower proportion of statin nonusers had a monthly income of NT$33,301 or more or resided in urban areas. Table 2 shows the lung cancer risk of the statin nonusers and users. After PS adjustment for age, sex, CCI, diabetes, hypertension, dyslipidemia, urbanization level, and monthly income, we analyzed the risk of lung cancer. The adjusted HRs (aHRs) of lung cancer were lower in the statin users than in the statin nonusers (aHR = 0.37, 95% confidence interval [CI]: 0.31 to 0.44). The stratified analysis showed that the aHRs were significantly lower in the statin users, particularly those aged 65–74 years, regardless of sex. Specifically, the aHRs of lung cancer were lower in the statin users than in the statin nonusers for every age group (40–64, 65–74, and ≥ 75 years; aHRs = 0.37, 0.31, and 0.43, respectively). The statin users also exhibited lower lung cancer aHRs than did the statin nonusers after sex stratification (women: aHR = 0.34, 95% CI: 0.25 to 0.45; men: aHR = 0.39, 95% CI: 0.32 to 0.48).

**Table 1:** Characteristics of the sample population

	Entire cohort (*n* = 43,802)		Patients using statins (≥ 28 cDDDs; *n* = 10,086)		Patients not using statins (< 28 cDDDs; *n* = 33,716)		*P*^a^
	*n*	%	*n*	%	*n*	%	
**Age, years (mean ± SD)**	62.92 (13.18)		61.55 (10.97)		63.33 (13.74)		< 0.001
40–54	14458	33.01	3180	31.53	11278	33.45	< 0.001
55–64	9644	22.02	2899	28.74	6745	20.01	
65–74	10455	23.87	2777	27.53	7678	22.77	
≥ 75	9245	21.11	1230	12.20	8015	23.77	
**Sex**							
Female	19715	45.01	5150	51.06	14565	43.20	< 0.001
Male	24087	54.99	4936	48.94	19151	56.80	
**CCI^+^**							
0	11279	25.75	2586	25.64	8693	25.78	< 0.001
1	12597	28.76	3014	29.88	9583	28.42	
2	9075	20.72	2195	21.76	6880	20.41	
≥ 3	10851	24.77	2291	22.71	8560	25.39	
**Diabetes**							
No	33491	76.46	6819	67.61	26672	79.11	< 0.001
Yes	10311	23.54	3267	32.39	7044	20.89	
**Hypertension**							
No	22067	50.38	4158	41.23	17909	53.12	< 0.001
Yes	21735	49.62	5928	58.77	15807	46.88	
**Dyslipidemia**							
No	31731	72.44	5785	57.36	25946	76.95	< 0.001
Yes	12071	27.56	4301	42.64	7770	23.05	
**Nonstatin lipid-lowering drugs**							
< 28 days	39267	89.65	7212	71.51	32055	95.07	< 0.001
28–365 days	3186	7.27	1923	19.07	1263	3.75	
> 365 days	1349	3.08	951	9.43	398	1.18	
**Metformin**							
< 28 days	35961	82.10	6286	62.32	29675	88.01	< 0.001
28–365 days	2684	6.13	964	9.56	1720	5.10	
> 365 days	5157	11.77	2836	28.12	2321	6.88	
**ACEI**							
< 28 days	23928	54.63	3066	30.40	20862	61.88	< 0.001
28–365 days	7925	18.09	1928	19.12	5997	17.79	
> 365 days	11949	27.28	5092	50.49	6857	20.34	
**Aspirin**							
< 28 days	28319	64.65	4161	41.26	24158	71.65	< 0.001
28–365 days	7385	16.86	2296	22.76	5089	15.09	
> 365 days	8098	18.49	3629	35.98	4469	13.25	
**Urbanization level**							
Urban	30539	69.72	7208	71.47	23331	69.20	< 0.001
Suburban	8914	20.35	1920	19.04	6994	20.74	
Rural	4349	9.93	958	9.50	3391	10.06	
**Monthly income (NT$)**							
0	3464	7.91	795	7.88	2669	7.92	< 0.001
1–21,000	15001	34.25	3067	30.41	11934	35.40	
21,000–33,300	12904	29.46	3165	31.38	9739	28.89	
≥ 33,301	12433	28.38	3059	30.33	9374	27.80	

a Comparison between statin use and no statin use.

+ CCI: Charlson comorbidity index.

**Table 2:** Risk of lung cancer in statin users and nonusers in the study cohort

Entire cohort (*n* = 43,802)	Patients not using statins (Total follow-up: 194,933.6 person-years)		Patients using statins (Total follow-up: 80,239.4 person-years)		aHR† (95% CI)
	No. of patients with lung cancer	Incidence rate (per 10^5^ person-years) (95% CI)	No. of patients with lung cancer	Incidence rate (per 10^5^ person-years) (95% CI)	
**Entire cohort**	1225	628.4 (593.2, 663.6)	159	198.2 (167.4, 229.0)	0.37 (0.31, 0.44)***
**Age, 40–64 years^a^**	419	360.5 (326.0, 395.0)	66	130.8 (99.2, 162.3)	0.37 (0.29, 0.49)***
**Age, 65–74 years^b^**	415	930.2 (840.7, 1019.7)	56	257.1 (189.8, 324.5)	0.31 (0.23, 0.41)***
**Age, ≥ 75 years^c^**	391	1146.9 (1033.2, 1260.6)	37	463.4 (314.1, 612.7)	0.43 (0.31, 0.61)***
**Female^d^**	361	413.1 (370.5, 455.7)	57	136.3 (100.9, 171.6)	0.34 (0.25, 0.45)***
**Male^e^**	864	803.4 (749.8, 857.0)	102	265.6 (214.0, 317.1)	0.39 (0.32, 0.48)***

a Total follow-up 116,228.5 person-year for patients not using statins and 50,476.0 for patients using statins.

b Total follow-up 44,612.9 person-year for patients not using statins and 21,778.3 for patients using statins.

c Total follow-up 34,092.2 person-year for patients not using statins and 7,985.1 for patients using statins.

d Total follow-up 87,389.9 person-year for patients not using statins and 41,828.7 for patients using statins.

e Total follow-up 107,543.7 person-year for patients not using statins and 38,410.7 for patients using statins.

CI: confidence interval.

aHR: adjusted hazard ratio.

† Main model was adjusted using propensity scores for age, sex, Charlson comorbidity index, diabetes, hypertension, dyslipidemia, urbanization level, and monthly income.

Statins dose-dependently reduced the risk of lung cancer in different cDDD subgroups; the main model was PS adjusted for age, sex, CCI, diabetes, hypertension, dyslipidemia, urbanization level, and monthly income (Table 3). Lipophilia statins comprised simvastatin, lovastatin, atorvastatin, and fluvastatin, whereas hydrophilia statins comprised pravastatin and rosuvastatin. Table 3 presents the lung cancer risk reduction demonstrated by lipophilia and hydrophilia statins in patients with COPD along with the doses and responses (*P* for trend < 0.001). Among individual statins, lovastatin and fluvastatin did not reduce the risk of lung cancer in patients with COPD significantly. The aHRs of lung cancer for patients using rosuvastatin, simvastatin, atorvastatin, and pravastatin were lower compared with that of statin nonusers (aHRs = 0.41, 0.44, 0.52 and 0.58, respectively). Our results revealed that individual statins reduced lung cancer risk at varying efficacies among COPD patients.

**Table 3:** Incidence rate and adjusted hrs of lung cancer associated with statin use during the follow-up period in COPD patients

Variable	No. of Patients	No. of Person-Years	No. of Patients With Lung cancer	Incidence Rate (per 105 person-years) (95% C.I.)	Adjusted HR (95% C.I.)	*P* for Trend
Total statin use						
Nonuser (< 28 cDDDs)	33716	194933.6	1225	628.4 (593.2, 663.6)	1.00	< 0.001
User (≥ 28 cDDDs)	10086	80239.4	159	198.2 (167.4, 229.0)	0.37 (0.31, 0.44)***	
28–90 cDDDs	2346	17095.6	49	286.6 (206.4, 366.9)	0.50 (0.38, 0.67)***	
91.365 cDDDs	3215	24193.1	57	235.6 (174.4, 296.8)	0.43 (0.33, 0.56)***	
> 365 cDDDs	4525	38950.7	53	136.1 (99.4, 172.7)	0.27 (0.20, 0.35)***	
Lipophilia statin use†						
Nonuser (< 28 cDDDs)	35008	204288.0	1248	610.9 (577.0, 644.8)	1.00	< 0.001
User (≤ 28 cDDDs)	8794	70885.0	136	191.9 (159.6, 224.1)	0.44 (0.37, 0.53)***	
28–90 cDDDs	2296	17069.8	46	269.5 (191.6, 347.4)	0.53 (0.40, 0.71)***	
91–365 cDDDs	3012	23258.7	47	202.1 (144.3, 259.8)	0.45 (0.34, 0.61)***	
> 365 cDDDs	3486	30556.4	43	140.7 (98.7, 182.8)	0.36 (0.26, 0.49)***	
Hydrophilia statin use‡						
Nonuser (< 28 cDDDs)	39878	242812.7	1339	551.5 (521.9, 581.0)	1.00	< 0.001
User (≤ 28 cDDDs)	3924	32360.4	45	139.1 (98.4, 179.7)	0.45 (0.33, 0.62)***	
28–90 cDDDs	1122	8876.1	18	202.8 (109.1, 296.5)	0.59 (0.37, 0.95)*	
91–365 cDDDs	1531	12432.2	13	104.6 (47.7, 161.4)	0.35 (0.20, 0.61)***	
> 365 cDDDs	1271	11052.0	14	126.7 (60.3, 193.0)	0.44 (0.26, 0.75)**	
Individual statin use (≤ 28 cDDDs)‡						
Simvastatin	3418	28625.0	37	129.3 (87.6, 170.9)	0.44 (0.31, 0.62)***	
Lovastatin	2109	18281.5	40	218.8 (151.0, 286.6)	0.74 (0.54, 1.03)	
Atorvastatin	5484	44678.1	81	181.3 (141.8, 220.8)	0.52 (0.41, 0.66)***	
Fluvastatin	1510	12855.7	27	210.0 (130.8, 289.2)	0.75 (0.51, 1.11)	
Pravastatin	1501	12654.5	19	150.1 (82.6, 217.7)	0.58 (0.36, 0.91)*	
Rosuvastatin	2741	22641.7	28	123.7 (77.9, 169.5)	0.41 (0.28, 0.59)***	

Main model is adjusted for age, sex, Charlson comorbidity index, diabetes, hypertension, dyslipidemia, level of urbanization, Monthly income in propensity score.

† Lipophilia statins include simvastatin, lovastatin, atorvastatin, and fluvastatin. Hydrophilia statins include pravastatin and rosuvastatin.

‡ The HRs of individual statin users (. 28 cDDDs) were compared with nonusers (< 28 cDDDs).

In the sensitivity analysis, PS adjustments were made to estimate the associations of age, sex, CCI, diabetes, hypertension, dyslipidemia, urbanization level, monthly income, and nonstatin lipid-lowering drugs, metformin, ACEI, and aspirin use with the incidence of lung cancer in different models. Table 4 shows that the effects of statins remained significant in the subgroups of various covariates when the main model was adjusted for PSs. Statins dose-dependently reduced the risk of lung cancer in all subgroups and the main model with additional covariates (nonstatin lipid-lowering drugs, metformin, ACEI, or aspirin use). All aHRs indicated that statins dose-dependently induced significant reductions in lung cancer risk in all subgroups, regardless of comorbidities or drug use (*P* < 0.001). Thus, our data revealed that statins show a dose-dependent chemopreventive effect against lung cancer.

**Table 4:** Sensitivity analysis of ahrs of statin use for reduction of lung cancer risk

	Statin use aHR (95% CI)				*P* for trend
	< 28 cDDDs	28–90 cDDDs	91–365 cDDDs	> 365 cDDDs	
**Main model†**	1.00	0.50 (0.38, 0.67)***	0.43 (0.33, 0.56)***	0.27 (0.20, 0.35)***	< 0.001
**Additional covariates‡**					
Main model + Nonstatin lipid-lowering drugs	1.00	0.52 (0.39, 0.69)***	0.46 (0.35, 0.60)***	0.29 (0.22, 0.38)***	< 0.001
Main model + Metformin	1.00	0.51 (0.38, 0.67)***	0.45 (0.34, 0.58)***	0.28 (0.21, 0.38)***	< 0.001
Main model + ACEI	1.00	0.52 (0.39, 0.69)***	0.48 (0.37, 0.63)***	0.33 (0.25, 0.43)***	< 0.001
Main model + Aspirin	1.00	0.52 (0.39, 0.69)***	0.46 (0.35, 0.61)***	0.30 (0.23, 0.40)***	< 0.001
**Subgroup effects**					
Age, years 40–64	1.00	0.62 (0.41, 0.94)*	0.41 (0.27, 0.64)***	0.23 (0.14, 0.36)***	< 0.001
65–74	1.00	0.33 (0.18, 0.58)***	0.45 (0.30, 0.67)***	0.22 (0.14, 0.35)***	< 0.001
≥ 75	1.00	0.59 (0.34, 1.03)	0.35 (0.19, 0.66)**	0.39 (0.23, 0.67)***	< 0.001
Sex					
Female	1.00	0.28 (0.15, 0.53)***	0.44 (0.29, 0.68)***	0.30 (0.20, 0.45)***	< 0.001
Male	1.00	0.64 (0.46, 0.88)**	0.43 (0.30, 0.60)***	0.24 (0.16, 0.35)***	< 0.001
CCI^+^					
0	1.00	0.47 (0.27, 0.84)*	0.32 (0.17, 0.58)***	0.29 (0.18, 0.49)***	< 0.001
1	1.00	0.52 (0.32, 0.87)*	0.53 (0.35, 0.82)**	0.21 (0.12, 0.37)***	< 0.001
2	1.00	0.44 (0.23, 0.83)*	0.59 (0.36, 0.97)*	0.28 (0.15, 0.50)***	< 0.001
≥ 3	1.00	0.53 (0.29, 0.98)*	0.23 (0.11, 0.48)***	0.25 (0.13, 0.46)***	< 0.001
Diabetes					
No	1.00	0.51 (0.37, 0.71)***	0.46 (0.34, 0.63)***	0.22 (0.16, 0.33)***	< 0.001
Yes	1.00	0.46 (0.25, 0.83)*	0.33 (0.20, 0.56)***	0.30 (0.20, 0.47)***	< 0.001
Dyslipidemia					
No	1.00	0.47 (0.33, 0.67)***	0.44 (0.32, 0.62)***	0.24 (0.16, 0.35)***	< 0.001
Yes	1.00	0.53 (0.33, 0.86)*	0.39 (0.25, 0.60)***	0.28 (0.19, 0.42)***	< 0.001
Hypertension					
No	1.00	0.50 (0.33, 0.75)***	0.50 (0.34, 0.73)***	0.22 (0.13, 0.36)***	< 0.001
Yes	1.00	0.50 (0.33, 0.74)***	0.37 (0.25, 0.53)***	0.27 (0.19, 0.38)***	< 0.001
Nonstatin lipid-lowering drugs					
< 28 days	1.00	0.53 (0.39, 0.73)***	0.42 (0.31, 0.58)***	0.25 (0.18, 0.35)***	< 0.001
28–365 days	1.00	0.49 (0.19, 1.26)	0.46 (0.22, 0.96)*	0.32 (0.16, 0.63)***	< 0.001
> 365 days	1.00	0.50 (0.06, 4.18)	1.47 (0.49, 4.38)	0.70 (0.24, 2.02)	0.644
Metformin					
< 28 days	1.00	0.53 (0.38, 0.72)***	0.42 (0.30, 0.58)***	0.27 (0.19, 0.38)***	< 0.001
28–365 days	1.00	0.29 (0.09, 0.93)*	0.28 (0.10, 0.78)*	0.25 (0.09, 0.69)**	< 0.001
> 365 days	1.00	0.74 (0.32, 1.71)	0.78 (0.44, 1.38)	0.38 (0.23, 0.65)***	0.001
ACEI					
< 28 days	1.00	0.56 (0.38, 0.84)**	0.44 (0.29, 0.68)***	0.21 (0.11, 0.41)***	< 0.001
28–365 days	1.00	0.53 (0.30, 0.93)*	0.68 (0.42, 1.10)	0.32 (0.16, 0.63)***	< 0.001
> 365 days	1.00	0.64 (0.35, 1.18)	0.56 (0.34, 0.91)*	0.51 (0.35, 0.74)***	< 0.001
Aspirin					
< 28 days	1.00	0.44 (0.29, 0.67)***	0.39 (0.26, 0.60)***	0.30 (0.19, 0.47)***	< 0.001
28–365 days	1.00	0.51 (0.29, 0.89)*	0.74 (0.47, 1.17)	0.19 (0.09, 0.44)***	< 0.001
> 365 days	1.00	1.13 (0.65, 1.97)	0.52 (0.30, 0.92)*	0.46 (0.30, 0.71)***	< 0.001

* *p* < 0.05

** *p* < 0.01

*** *p* < 0.001.

a HR: adjusted hazard ratio.

+ CCI: Charlson comorbidity index.

† Main model was adjusted using propensity scores for age, sex, Charlson comorbidity index, diabetes, hypertension, dyslipidemia, urbanization level, and monthly income.

‡ Models were adjusted for covariates in the main model as well as each additional listed covariate.

## DISCUSSION

Recently, interest in the function of systemic inflammation in COPD has been increasing [23–27]. Epidemiological studies have shown that elevated levels of systemic inflammatory markers, particularly C-reactive protein (CRP), interleukin 6 (IL-6), and fibrinogen, predict poor outcomes in COPD, including accelerated loss of lung function, greater propensity for infective exacerbations, and greater mortality [28–30]. This systemic inflammation has three likely mechanisms. The first is a “spillover” effect from inflammation (driven primarily in the lungs in response to aeropollutants, mainly cigarette smoke) to neutrophilic inflammation and finally to recurrent infection [31, 32]. The second is the existence of an inherent systemic-based proinflammatory state conferred by a genetic disposition [23, 33, 34]. Smoking, as a recurring proinflammatory stimulus to the pulmonary and immune systems, considerably enhances this inflammatory disposition. The final possible mechanism is elevated systemic inflammation, which has been linked to progressive loss of lung function [24–27, 35–37] and to many types of cancer [37–39].

CRP is mainly a marker of inflammation. When some organs are chronically inflamed, they are at greater cancer risk [40, 41]. Increased CRP levels are associated with increased cancer risk [42]. A large-scale prospective study reported the effects of statins on mortality in patients with COPD by using the Rotterdam study data; stratification by high-sensitivity CRP revealed that all-cause mortality was 78% lower among patients with CRP ≥ 3 mg/L, whereas it was only by 21% lower among those with CRP < 3 mg/L [43]. The authors concluded that statins therapy primarily benefited the all-cause mortality of patients whose CRP levels indicated underlying systemic inflammation [43].

Statins attenuate both pulmonary and systemic inflammation through their effects on the NF-κB/STAT3 proinflammatory pathways [23]. Statins are considered effective anti-inflammatory agents that reduce the levels of systemic markers (IL-6 and CRP) by more than 50% in a few days [44]. Statins exhibit immune-modulating (i.e., anti-inflammatory) effects that may be particularly crucial in COPD, in which both pulmonary and systemic inflammation are believed to be central causes of symptoms (exertional breathlessness, cough, and fatigue), hospitalization, and premature death (from pulmonary infection or exacerbation, lung cancer, and cardiac disease). Therefore, a great need exists for novel COPD treatments that minimize neutrophil-driven pulmonary and systemic inflammation that alters the natural history of the disease by slowing lung function decline, minimizing cardiovascular and respiratory infection-related morbidities, and reducing cancer risk [23]. A meta-analysis showed no effect statin use on the risk of lung cancer [17]; nevertheless, in the present study, COPD patients with a high risk of lung cancer who used statins exhibited a 63% reduced lung cancer risk (Table 2). This is the first study to report that statin-based agents could be of chemopreventive value against lung cancer, specifically for patients with COPD.

Rosuvastatin, atorvastatin, and simvastatin cause the greatest percentage change in LDL-C; thus, they are preferred for use in patients who require a potent statin because of high cardiovascular risk or who require a > 35% reduction in LDL-C level. Rosuvastatin is relatively more potent than atorvastatin [45, 46] and both are significantly more potent than simvastatin, lovastatin, pravastatin, or fluvastatin [46, 47]. At their maximal prescribed doses, rosuvastatin and atorvastatin cause LDL-C level reductions greater than those caused by other available statins. Statin therapy typically increases HDL-C levels; however, these effects vary depending on the statin type and are not correlated with the effects on LDL-C levels. For example, simvastatin and rosuvastatin increase HDL-C levels as their doses are increased, whereas at higher doses, atorvastatin attenuates increases in HDL-C levels [48]. Atorvastatin and rosuvastatin are more effective for reducing triglyceride levels in patients with hypercholesterolemia than other statins are [46, 49–51]. Our results revealed that different statins were associated with varying reductions in lung cancer risk among the COPD patients (Table 3). Notably, the stronger efficacies of rosuvastatin, atorvastatin, and simvastatin in reducing LDL-C and triglyceride levels and increasing high HDL-C levels were proportional to the decreased aHRs of lung cancer risk (Table 3). No clear data regarding the use of different individual statins has been previously reported [17]. In our study, lovastatin and fluvastatin exhibited no significant reduction in lung cancer risk in patients with COPD. We are the first to report that rosuvastatin, atorvastatin, and simvastatin show stronger chemopreventive effect against lung cancer risk in patients with COPD. Of these, rosuvastatin exhibited the highest chemopreventive potential, followed by simvastatin and atorvastatin.

Statin use dose-dependently reduced lung cancer risk in the COPD patients and in the main model with additional covariates (Table 4). The use of aspirin, nonstatins lipid-lowering drugs, metformin, and ACEI also has an anticancer effect [5]. When the cDDDs of aspirin, metformin, and ACEI were > 365, the chemopreventive effect of statins against lung cancer was masked (Table 4). However, our sensitivity analysis indicated that when the cDDDs of statins increased to > 365, the aHRs of lung cancer risk in the COPD patients decreased significantly. However, the aHRs of lung cancer risk were nonsignificant when the cDDDs of nonstatin lipid-lowering drugs were > 365 (Table 4). These outcomes might explain the independent chemopreventive effects of aspirin, metformin, ACEI, and statins. However, unknown associations between nonstatin lipid-lowering drugs and statins were observed in the reduction of lung cancer risk in the COPD patients. This study is also the first report that statins exert dose–response and chemopreventive effects against lung cancer in patients with COPD.

However, this study has potential limitations. The biases of additional risk factors associated with COPD and lung cancer, including indoor and outdoor air pollution, domestic use of biomass fuels, occupational exposure to dust and fumes, and smoking could not be eliminated [52, 53]. A future large-scale randomized trial with a suitable regimen in well-selected patients must compare standard approaches to obtain this crucial information. However, methodological issues may obscure the precise relationship between these factors and lung cancer risk. According to one theory, higher urbanization levels and income are associated with lower lung cancer risk. In our study, we used PSs to match age, sex, CCI, diabetes, hypertension, dyslipidemia, urbanization level, and monthly income. Urbanization level and monthly income are nonvalidated alternatives to lifestyle factors and environmental levels. To obtain more appropriate information, a large-scale randomized trial should apply a suitable regimen to appropriately selected patients for comparing standard approaches. Moreover, in this study, the diagnoses of lung cancer and all other comorbidities were completely dependent on ICD codes. However, the NHI Administration randomly reviews medical records and interviews patients to validate diagnoses. Hospitals with outlier diagnoses and practices may be audited and penalized heavily if malpractice or discrepancies are discovered. Another limitation is that information regarding several unmeasured confounders, including body mass index, smoking, alcohol intake, and use of other over-the-counter drugs (some of which are associated with lung cancer), is unavailable in the NHIRD. However, considering the magnitude and significance of the observed effects, it is unlikely that these limitations compromised the results. Finally, this was not a prospective randomized blinded study; hence, a cause–effect relationship could not be established. The findings of this study suggest that statins dose-dependently exert a significant chemopreventive effect against lung cancer in COPD patients. Additional randomized studies are required to verify these findings.

## MATERIALS AND METHODS

The National Health Insurance (NHI) program, which was established in 1995, currently provides comprehensive health insurance coverage to 98% of the more than 23 million people in Taiwan. In this study, we used data from the National Health Insurance Research Database (NHIRD). No statistically significant differences were observed in age, sex, or health care costs between the NHIRD sample group and all NHI enrollees. Data that could be used to identify patients or care providers, including medical institutions and physicians, are encrypted before being sent to the National Health Research Institutes for construction of the NHIRD. The Institutes further encrypts the data before being releasing the database to researchers. Theoretically, the NHIRD data alone is insufficient to identify any individual. All researchers using the NHIRD and its data subsets must sign a written agreement declaring that they have no intention of attempting to obtain information that could potentially violate the privacy of patients or care providers [5].

Our study cohort comprised all patients diagnosed with COPD (according to International Classification of Diseases, Ninth Revision, Clinical Modification [ICD-9-CM] codes) at health care facilities in Taiwan (*n* = 116,017) between January 1, 2001 and December 31, 2012. We excluded patients without a subsequent outpatient visit, emergency department visit, or inpatient hospitalization for COPD within 12 months of the first presentation (*n* = 48,212); these patients were considered to not have COPD (Figure 1). We also excluded 15,436 patients who were younger than 40 years old (*n* = 52,369) and had any inpatient or outpatient diagnosis related to cancer before the enrollment date (*n* = 5,353) or had any statin prescribed within 6 months before the index date (*n* = 3,214).

**Figure 1:** Patient selection flowchart

Our final study cohort contained 43,802 patients diagnosed with COPD in Taiwan over the 11-year period, 10,086 of whom used statins and 33,716 of whom did not. Each patient was followed to assess lung cancer risk or protective factors. In addition, we considered the demographic characteristics of age and sex; comorbidities of diabetes, hypertension, dyslipidemia, and Charlson comorbidity index (CCI); urbanization level; monthly income; and use of nonstatin lipid-lowering drugs, metformin, aspirin, and angiotensin-converting enzyme inhibitor (ACEI). The index date of statin use was the date of COPD confirmation. Because we aimed to evaluate the preventive effects of statin use in COPD patients who have a high lung cancer risk, the primary endpoint was lung cancer risk and the secondary endpoints were different benefits if different doses or types of statins used. The defined daily dose (DDD)—recommended by the World Health Organization—is a measure of the prescribed drug amount. DDD is the assumed average maintenance dose per day of a drug consumed for its main indication in adults.^12^ To examine the dose–response relationship, we categorized statin use into four groups in each cohort (< 28, 28–90, 91–365, and > 365 cumulative DDDs [cDDDs]) because the duration of the refill card was 3 months. Patients receiving < 28 cDDDs were defined as nonstatin users (Tables 2–4) [54]. Furthermore, to examine the preventive effect of different types of statins, we categorized statin use into different individual statin use groups in each cohort (Table 3).

Propensity scores (PSs) were derived using a logistic regression model to estimate the effect of statins by accounting for the covariates predicting receiving the intervention (statins). This method is commonly used in observational studies to reduce selection bias [55]. The covariates in the main model were PS adjusted for age, sex, CCI, diabetes, hypertension, dyslipidemia, urbanization level, and monthly income in New Taiwan dollars (NT$0, NT$1–21,000, NT$21,000–33,300; and ≥ NT$33,301) (Table 2). The endpoint for both statin users and nonusers was the diagnosis of lung cancer (ICD-9-CM 162) with a subsequent outpatient visit, emergency department visit, or inpatient hospitalization for lung cancer within 12 months of diagnosis; the nonusers were used as the reference arm. The cumulative incidence of lung cancer in the two groups was estimated using the Kaplan–Meier method.

A time-dependent Cox proportional hazard model was used to calculate the hazard ratios (HRs) of lung cancer in the statin users and nonusers. The HRs were adjusted for age, sex, CCI, diabetes, hypertension, dyslipidemia, urbanization level, and monthly income in the multivariate analysis. A stratified analysis was conducted to evaluate the effect of statin use on age and sex (Table 2). All analyses were conducted using SAS software (Version 9.3; SAS, Cary, NC, USA); two-tailed *P* < 0.05 was considered significant. In sensitivity analyses, external adjustments are used to improve the understanding of the effects of drugs and other covariates in epidemiological database studies [56]. Hence, in our sensitivity analyses, data were adjusted in different models to estimate the association of lung cancer incidence with age, sex, diabetes, dyslipidemia, hypertension, CCI, anxiety disorder, and the use of nonstatin lipid-lowering drugs, metformin, aspirin, and ACEI. The drug use-stratified models were adjusted for covariates in the main model and for each additional covariate (Table 4).

## CONCLUSIONS

Statins dose-dependently exert a significant chemopreventive effect against lung cancer in COPD patients. Rosuvastatin shows the highest chemopreventive potential, followed by simvastatin and atorvastatin.
